The article "LncRNA TUBA4B functions as a competitive endogenous RNA to inhibit gastric cancer progression by elevating PTEN via sponging miR-214 and miR-216a/b" was retracted in 2022. Reasons: results that could not be reproduced; contaminated cell lines or tissues; errors in the data; unreliable results or conclusions.

# LncRNA TUBA4B functions as a competitive endogenous RNA to inhibit gastric cancer progression by elevating PTEN via sponging miR-214 and miR-216a/b

**DOI:** 10.1186/s12935-019-0879-x

**Published:** 2019-06-07

**Authors:** Jianbo Guo, Yan Li, He Duan, Lu Yuan

**Affiliations:** Department of General Surgery, The Fourth Affiliated Hospital of China Medical University, 4 Chongshan East Street, Shenyang, 110032 Liaoning People’s Republic of China

**Keywords:** Long non-coding RNA, TUBA4B, Gastric cancer, ceRNA, PI3K/AKT signaling, Biomarker

## Abstract

**Background:**

Emerging evidence demonstrates that long non-coding RNA (lncRNA) is an important regulator in tumorigenesis and development. Tubulin Alpha 4B (TUBA4B), a novel lncRNA, was recently proposed as a tumor suppressor in several human cancers. However, its role in gastric cancer (GC) remains unclear. In this study, we aimed to investigate the expression level, clinical implication, biological function and potential regulatory mechanism of TUBA4B in GC.

**Methods:**

qRT-PCR was employed to detect the expression of TUBA4B in GC tissues, cell lines and plasma. In vitro and in vivo experiments were carried out using colony formation/CCK-8/transwell invasion/cell apoptosis assay and xenograft tumor model, respectively. mRNA sequencing was used to identify the TUBA4B-related downstream genes.

**Results:**

TUBA4B was significantly decreased in GC tissues, cells and plasma. Low TUBA4B was positively correlated with larger tumor size, lymph node metastasis and advanced TNM stage. Moreover, TUBA4B was identified as an effective biomarker for the diagnosis and prognosis of patients with GC. Functionally, ectopic expression of TUBA4B inhibited GC cell proliferation, invasion and induced apoptosis in vitro as well as dampened tumor growth and metastasis in vivo. Furthermore, TUBA4B was found to be a competitive endogenous RNA (ceRNA) that could physically bind to and sequester miR-214 and miR-216a/b to increase the expression of their common downstream target PTEN, resulting in inactivation of PI3K/AKT signaling pathway, thereby retarding GC progression.

**Conclusion:**

Our data highlight the compelling regulatory role of TUBA4B in GC, and reactivation of TUBA4B may be a promising therapeutic avenue for GC patients.

**Electronic supplementary material:**

The online version of this article (10.1186/s12935-019-0879-x) contains supplementary material, which is available to authorized users.

## Background

Gastric cancer (GC) is the fifth most frequently diagnosed cancer and the third leading cause of cancer-associated death worldwide, with more than 1 million new cases and an estimated 783,000 deaths in 2018 [1]. GC is an extremely complicated disease with a large number of genetic and epigenetic changes. Despite extensive studies on the pathogenesis of GC in recent decades, the 5-year survival rate of GC remains poor, mainly due to the lack of effective biomarkers for diagnosis of early GC as well as local recurrence and metastasis after operation [2]. Therefore, continued research into this field is urgently needed to discover novel and more effective biomarkers and therapeutic targets for GC.

Long non-coding RNA (lncRNA) is a type of RNA molecule with a transcript length of more than 200 nucleotides and lacks protein-coding potential [3]. Initially, lncRNA was regarded as the “garbage” of genome transcription without biological function. Nevertheless, recent studies have shown that lncRNA is involved in various important regulatory processes, such as X chromosome silencing, genomic imprinting, chromatin modification, transcriptional activation, transcriptional interference, intranuclear transport and so on [4]. The transcripts generated by 4% to 9% of the mammalian genome sequence are lncRNAs (the corresponding protein-encoding RNA is 1%) [5]. Although the research on lncRNA has progressed rapidly in recent years, the biological functions of most lncRNAs remain largely unknown.

It is well documented that lncRNA is able to tightly regulate gene expression at transcriptional and post-transcriptional levels, which makes it closely related to tumorigenesis and development [6]. The most widely studied role of lncRNA is that it is capable of functioning as a competitive endogenous RNA (ceRNA) that interacts with and sequesters miRNAs to alleviate the repression of miRNAs on target mRNAs [7]. For example, Chen et al. [8] reported that lncRNA ZFAS1 contributed to the progression of colorectal cancer by sponging miR-150-5p to upregulating VEGFA expression. LncRNA CASC2 was proposed to increase PTEN expression via abundantly sponging miR-21 to inhibit pancreatic carcinoma malignancy [9]. LncRNA CAR10 was found to promote lung adenocarcinoma metastasis by directly binding with and inhibiting miR-30/203 to elevate the expression of SNAI family [10]. These studies suggest that the ceRNA network plays a vital regulatory role in tumorigenesis and aggressiveness.

Recently, a novel lncRNA, Tubulin Alpha 4B (TUBA4B), has been identified as an important tumor suppressor in various human cancers [11]. However, its role in GC remains unexplored. In the present study, we aimed to investigate the expression level, clinical implication, biological function and potential regulatory mechanism of TUBA4B in GC.

## Materials and methods

### Tissues, cell lines and plasma

A total of 83 fresh GC and paired normal tissues were obtained from The Fourth Affiliated Hospital of China Medical University. These tissues were accurately diagnosed as GC by two experienced pathologists and then placed into liquid nitrogen to protect RNA integrity. To assess the diagnostic value of TUBA4B, we also collected plasma samples from GC patients (n = 37) and healthy controls (n = 37). This study was conducted with the approval of the ethics committee of China Medical University. All participants enrolled in this study had signed the informed consent.

To explore the biological function of TUBA4B, a human gastric epithelial GES-1 cells and five GC cell lines (AGS, SGC-7901, BGC-823, MGC-803 and HGC-27) were used. All cells were purchased from ATCC and cultured in DMEM medium with 10% fetal bovine serum. Mycoplasma test was performed on each cell line every 3 months.

### Quantitative reverse transcription polymerase chain reaction (qRT-PCR)

TRIzol reagent (Invitrogen, CA, USA) was employed to extract total RNA from GC tissues, cell lines and plasma. RNA quantification was performed using SYBR Green SuperMix (Roche, Basel, Switzerland) as per manufacturer’s protocols. GAPDH and U3 were used as the internal control for lncRNA/mRNA and miRNAs, respectively. The primer sequences are as follows:

TUBA4B: Forward (5′ to 3′)-CCCACAGGCTTTAAGGTTGA;
  Reverse (5′ to 3′)-AGGCCATAGTGATGGCTGTC
miR-214: Forward (5′ to 3′)-TGCCTGTCTACACTTGCT;
  Reverse (5′ to 3′)-GTCCAGTTTTTTTTTTTTTTTGCAC
mir-216a: Forward (5′ to 3′)-GCAGTAATCTCAGCTGGCA;
  Reverse (5′ to 3′)-TCCAGTTTTTTTTTTTTTTTCACAGT
mir-216b: Forward (5′ to 3′)-GCAGAAATCTCTGCAGGCA;
  Reverse (5′ to 3′)-GGTCCAGTTTTTTTTTTTTTTTCAC
GAPDH: Forward (5′ to 3′)-TGCACCACCAACTGCTTAGC;
  Reverse (5′ to 3′)-GGCATGGACTGTGGTCATGAG
U3: Forward (5′ to 3′)-TTCTCTGAGCGTGTAGAGCACCGA;
  Reverse (5′ to 3′)-GATCATCAATGGCTGACGGCAGTT

### Establishment of stable TUBA4B overexpression GC cell lines

The full-length sequence of TUBA4B was synthesized and inserted into pLenti-GIII-CMV-GFP-2A-Puro vector (Applied Biological Materials, BC, Canada), followed by package into lentiviral particles using Lentifectin™ solution (Applied Biological Materials) for high efficiency transduction and stably integrated expression. Next, MGC-803 and HGC-27 cells were transducted with above lentiviral vector at a multiplicity of infection of 25. Two days later, cells were treated with 1.2 μg/mL puromycin (Applied Biological Materials) to select stable TUBA4B overexpression GC cell lines. The overexpression efficiency was determined by qRT-PCR analysis.

### Cell proliferation and apoptosis assays

Cell Counting Kit-8 (CCK-8) and colony formation assays were utilized to measure the proliferative ability of MGC-803 and HGC-27 cells after TUBA4B overexpression. For CCK-8 assay, cells with or without TUBA4B overexpression were plated into 96-well plates and then incubated with 10 μL CCK-8 reagent (Sangon Biotech, Shanghai, China), followed by analysis of absorbance. For colony formation assay, MGC-803 and HGC-27 cells with or without TUBA4B overexpression were plated into 6-well plates. After 14 days, cells were fixed by methanol and stained by crystal violet. Cell apoptosis was carried out using Annexin V/7-AAD staining kit (Sino Biological Inc., Beijing, China) as per the standard protocol.

### Transwell invasion assay

The invasive ability of GC cells was conducted using the Boyden chambers containing 24-well transwell plates (BD Inc., USA) with 8 mm pore size. MGC-803 and HGC-27 cells were seeded into on the upper surface of the chambers and DMEM medium containing 10% fetal bovine serum was added into the 24-well transwell plates. 18 h later, the invaded cells on the lower surface of the chambers were washed, fixed and stained.

### Animal study

To evaluate the effect of TUBA4B on in vivo tumor growth, 5 × 10^6^ control or TUBA4B-overexpressing MGC-803 cells were subcutaneously into the axilla of nude mice (n = 10 in each group), the volume measurement of subcutaneous tumors in each nude mice was conducted every 5 days. On the 30th day, all nude mice were euthanized and the tumors were dissected and weighed. To test the effect of TUBA4B on in vivo tumor metastasis, 1 × 10^6^ control or TUBA4B-overexpressing MGC-803 cells were injected into the nude mice (n = 8 in each group) through the tail vein. Monitoring of lung metastasis was carried out using the IVIS Lumina II system. Five weeks later, all nude mice were sacrificed and the lungs were dissected and metastatic nodules were calculated, followed by H&E staining. All nude mice used were purchased from Shanghai Laboratory Animal Center (Shanghai, China) and grown under specific-pathogen-free condition. The animal study was approved by the Animal Policy and Welfare Committee of China Medical University.

### mRNA sequencing

Total RNA from control or TUBA4B-overexpressing MGC-803 cells was extracted by TRIzol reagent (Invitrogen) and subjected to mRNA sequencing. The high-throughput sequencing and subsequent data analysis was performed by GENESKY company (Shanghai, China) using the standard BGISEQ-500 platform. A total of 17,768 genes were detected. The value of differentially expressed mRNA after TUBA4B overexpression was set with fold change ≥ 2 and *p *< 0.05. Then, the Kyoto Encyclopedia of Genes and Genomes (KEGG) pathway and Gene Set Enrichment Analysis (GSEA) were conducted using DAVID v6.8 and GSEA v3.0 software, respectively.

### Western blot

Total protein from control or TUBA4B-overexpressing MGC-803 and HGC-27 cells was isolated using 100 μL RIPA lysis buffer and subjected to protein quantification with BCA Protein Assay Kit (Sangon Biotech). Next, the protein was separated on 10% SDS-PAGE gel and **t**hen transferred onto PVDF membrane, followed by blockade with 5% dried skimmed milk or bovine serum albumin (for p-PI3K and p-AKT) and incubation with corresponding primary and secondary antibodies. Lastly, the membrane was strictly washed by tris buffered saline tween (TBST) and visualized by ECL western blotting substrate (Invitrogen). The primary antibodies used in this study are as following: anti-PTEN (#22034-1-AP, Proteintech, IL, USA), anti-p-PI3K (#4228, CST, MA, USA), anti-PI3K (#4249, CST), anti-p-AKT (#4060, CST), anti-AKT (#2920, CST), anti-GAPDH (#10494-1-AP, Proteintech).

### Biotin pull-down assay

Total protein from MGC-803 and HGC-27 cells were obtained through using lysis buffer and then incubated with control or TUBA4B probe labeled with biotin at 4 °C overnight, followed by incubation with streptavidin-coupled magnetic beads (Invitrogen) on the next day at 25 °C for 2 h. Then, the TUBA4B binding miRNAs were washed and eluted and detected by qRT-PCR analysis.

### Luciferase reporter assay

The full-length sequences of TUBA4B and PTEN 3′-UTR with putative wild-type or mutant miR-214/216a/b binding sites were embedded into FL reporter vector (Obio, Shanghai, China), respectively. MGC-803 and HGC-27 cells were seeded into 96-well plates and then co-transfected with a mixture of 5 pmol miR-214/216a/b mimics, 50 ng above FL reporter vectors and 5 ng pRL-CMV Renilla luciferase reporter vectors using Lipofectamine 3000 (Invitrogen). After 2 days of co-transfection, the luciferase activity was detected using Amplite Luciferase Reporter Gene Assay Kit (AAT Bioquest, CA, USA) as per manufacturer’s protocol.

### Statistical analysis

Data were shown as mean ± standard deviation (SD) representing at least three effective independent replicates. The differences between groups were analyzed by Student’s t or Chi-square test. The value of TUBA4B in diagnosis and prognosis of GC was assessed by receiver operating characteristic (ROC) curve and Kaplan–Meier plot, respectively. All statistical results were two-tailed and produced by Graphpad 8.0 software. *p* < 0.05 was considered to be significant.

## Results

### TUBA4B is decreased in GC tissues, cells and plasma

First, we collected 83 pairs of GC and adjacent normal tissues to test TUBA4B expression. The qRT-PCR results showed that TUBA4B was dramatically downregulated in GC tissues compared with para-carcinoma tissues (Fig. 1a). Consistently, low TUBA4B expression was also pervasively observed in five GC cell lines (Fig. 1b). Additionally, we also detected the expression level of plasma TUBA4B, as shown in Fig. 1c, plasma TUBA4B was significantly lower in GC patients than that in healthy controls. And ROC curve was plotted based on plasma TUBA4B expression level (Fig. 1d), the results displayed that the area under curve (AUC) was 0.8075 (95% CI 0.7103 to 0.9047), implying that plasma TUBA4B was an effective diagnostic biomarker for GC. Moreover, TUBA4B downregulation was closely associated with larger tumor size, lymph node metastasis and advanced TNM stage (Table 1). Importantly, GC patients with low TUBA4B expression had shorter survival time than those with high TUBA4B expression (Fig. 1e), and this result was also confirmed by the survival data of GC patients from TCGA database (Fig. 1f). Besides, we performed uni- and multivariate analysis for evaluating prognostic predictors of GC patients, the results revealed that TNM stage and lymph node metastasis were independent risk prognostic factors, whereas TUBA4B was an independent protective prognostic factor (Table 2). Taken together, these data suggest that loss of TUBA4B is an early process of GC, which may play an important role in GC tumorigenesis.

**Fig. 1:** Low TUBA4B is identified in GC and its downregulation predicts poor outcome. **a** qRT-PCR analysis of TUBA4B expression in 83 pairs of GC and adjacent normal tissues. **b** qRT-PCR analysis of TUBA4B expression in the human gastric epithelial GES-1 cells and five GC cell lines. **c** qRT-PCR analysis of TUBA4B expression in plasma samples from GC patients (n = 37) and healthy controls (n = 37). **d** The ROC curve for evaluating the prognostic value of plasma TUBA4B expression in GC. **e**, **f** The Kaplan–Meier survival curve of GC patients with low and high TUBA4B expression in our study or in TCGA database. *p < 0.05, **p < 0.01, ***p < 0.001

**Table 1:** Correlation between TUBA4B expression and clinicopathological features in GC patients (n = 83)

Parameters	All cases	TUBA4B expression		*p* value
		Low (n = 42)	High (n = 41)	
Gender				
Male	63	31	32	0.652
Female	20	11	9	
Age (years)				
≤ 60	31	17	14	0.551
> 60	52	25	27	
Tumor size				
≤ 5	45	18	27	*0.036*
> 5	38	24	14	
Lymph node metastasis				
No	39	13	26	*0.003*
Yes	44	29	15	
TNM stage				
I–II	36	11	25	*0.001*
III–IV	47	31	16	
Differentiation grade				
Well/moderate	43	19	24	0.225
Poor	40	23	17	

TNM stage was based on the 8th edition American Joint Committee on Cancer (AJCC) staging

Italic values indicate significance of *p* value (*p* < 0.05)

**Table 2:** Uni- and multivariate analysis of prognostic predictors in GC patients (n = 83)

Variable	Univariate analysis		Multivariate analysis	
	HR (95% CI)	*p* value	HR (95% CI)	*p* value
Gender (male)	1.089 (0.635–1.456)	0.752		
Age (> 60)	1.022 (0.574–1.265)	0.637		
Tumor size (> 5)	1.95 (1.152–3.867)	*0.034*	1.21 (0.845–3.25)	0.568
Lymph node metastasis (yes)	3.41 (1.82–5.66)	*0.002*	2.67 (1.24–4.35)	*0.031*
TNM stage (III–IV)	5.361 (2.964–9.476)	< *0.001*	3.954 (2.241–6.893)	*0.025*
Differentiation (poor)	1.43 (0.681–2.24)	0.432		
TUBA4B (high)	0.542 (0.225–0.813)	< *0.001*	0.612 (0.286–0.842)	*0.016*

Italic values indicate significance of *p* value (*p* < 0.05)

### Overexpression of TUBA4B inhibits GC cell proliferation and invasion both in vitro and in vivo

To determine the biological function of TUBA4B in GC, we stably overexpressed TUBA4B in MGC-803 and HGC-27 cells using lentivirus vectors (Fig. 2a). CCK-8 and colony formation assays showed that the proliferative capabilities of MGC-803 and HGC-27 cells were substantially attenuated after exogenous TUBA4B expression (Fig. 2b–d). Similarly, overexpression of TUBA4B reduced the invasive abilities of cells by nearly 50% (Fig. 2e). And flow cytometry apoptotic analysis revealed that TUBA4B-overexpressing MGC-803 and HGC-27 cells arose more apoptosis than control cells (Fig. 2f). Further, we established the subcutaneous xenograft (n = 10 per group) and experimental lung metastasis (n = 8 per group) models to assess the effects of TUBA4B on GC cell proliferation and invasion in vivo, respectively. The results showed that enforced expression of TUBA4B resulted in smaller tumors and fewer lung metastatic nodules (Fig. 2g–i). Overall, these above functional experiments indicate that TUBA4B is a negative regulator of GC aggressive phenotype.

**Fig. 2:** Enforced expression of TUBA4B impedes GC aggressive phenotype both in vitro and in vivo. **a** qRT-PCR analysis of TUBA4B expression in TUBA4B-overexpressing MGC-803 and HGC-27 cells. **b**–**d** CCK-8 and colony formation assays for testing the proliferative abilities of MGC-803 and HGC-27 cells with or without TUBA4B overexpression. **e** Transwell assay using chamber coated with matrigel for assessing the invasive capabilities of MGC-803 and HGC-27 cells with or without TUBA4B overexpression. **f** Annexin V and 7-AAD double staining for detecting the apoptotic rate in MGC-803 and HGC-27 cells with or without TUBA4B overexpression. **g** Representative image showing subcutaneous tumors of nude mice in the indicated two groups, as well as the statistical results of the volume and weight of tumors. **h**, **i** Representative images showing lung metastasis in the indicated two groups monitored by IVIS Lumina II system and H&E staining. *p < 0.05, **p < 0.01, ***p < 0.001

### TUBA4B functions through regulation of PTEN/PI3K/AKT signaling

To explore the potential mechanism by which TUBA4B impedes GC progression, we performed mRNA sequencing in control and TUBA4B-overexpressing MGC-803 cells. We found a large number of differentially expressed genes (fold change ≥ 2 and *p *< 0.05) after TUBA4B overexpression (Fig. 3a). KEGG pathway and GSEA analysis displayed that TUBA4B expression was strongly negatively correlated with PI3K/AKT signaling (Fig. 3b, c). Given that PTEN, a well-known suppressor of PI3K/AKT signaling [12], was notably upregulated in TUBA4B-overexpressing MGC-803 cells (Fig. 3a), we thus inferred that TUBA4B was able to dampen PI3K/AKT signaling via elevating PTEN, leading to inhibiting GC progression. As expected, western blot results showed that PTEN was markedly increased, while p-PI3K and p-AKT were dramatically decreased in MGC-803 and HGC-27 cells overexpressing TUBA4B in comparison to control cells (Fig. 3d, e). Furthermore, we found that the weakened cell malignant phenotype induced by TUBA4B was evidently rescued after transfection with small interfering RNA against PTEN or constitutively-activated Akt1 (myr-AKT) vector (Fig. 3f–h). In all, these findings demonstrate that the PTEN/PI3K/AKT signaling pathway is involved in the process of TUBA4B tumor suppression.

**Fig. 3:** TUBA4B inhibits the oncogenic PI3K/AKT pathway via upregulation of PTEN. **a** The hierarchical clustering map showing the differentially expressed genes after TUBA4B overexpression. **b** Kyoto Encyclopedia of Genes and Genomes (KEGG) pathway analysis of the differentially expressed genes after TUBA4B overexpression. **c** Gene Set Enrichment Analysis (GSEA) showing the negative correlation between TUBA4B and PI3K/AKT pathway. **d**, **e** Western blot analysis of the indicated protein expression in TUBA4B-overexpressing MGC-803 and HGC-27 cells. **f**–**h**. CCK-8 proliferative, transwell invasion and cell apoptosis assays in TUBA4B-overexpressing MGC-803 and HGC-27 cells after transfected with PTEN siRNA or constitutively-activated Akt1 (myr-AKT) vector. **p < 0.01, ***p < 0.001

### TUBA4B physically interacts with miR-214 and miR-216a/bp

Next, we wondered how TUBA4B regulates the expression level of PTEN. We first determined the subcellular localization of TUBA4B, the qRT-PCR and FISH results showed that TUBA4B preferentially localized in the cytoplasm (Fig. 4a, Additional file 1: Figure S1). It has been reported that cytoplasmic lncRNA functioned mainly via sponging miRNAs [13]. We then searched for potential TUBA4B-binding miRNAs using miRCode database (http://www.mircode.org/), besides, we also utilized miRWalk database to search for miRNAs that might bind to the 3′-UTR of PTEN. As shown in Fig. 4b, eight miRNAs were predicted to be involved in TUBA4B-mediated PTEN regulation. To valid this prediction, RNA pull-down assay was carried out using biotin-labeled probe. The results showed that miR-214 and miR-216a/b, but not the other five miRNAs, were abundantly enriched by TUBA4B probe in comparison to control probe both in MGC-803 and HGC-27 cells (Fig. 4c). Moreover, luciferase reporter assay revealed that overexpressed miR-214 or miR-216a/b could not inhibit the luciferase activity of TUBA4B reporter vector containing mutant miR-214 or miR-216a/b binding site, whereas dramatically attenuated the luciferase activity of wild-type one (Fig. 4d–f). In addition, we found that the expression levels of miR-214 and miR-216a/b were significantly downregulated in MGC-803 and HGC-27 cells overexpressing TUBA4B (Fig. 4g), and this phenomenon was also observed in the xenograft tumor model (Fig. 4h). Importantly, the survival data from Kaplan–Meier plotter (http://kmplot.com/analysis/) showed that GC patients with high miR-214 or miR-216a/b expression had worse prognosis than those with low miR-214 or miR-216a/b expression (Fig. 4i). Collectively, these results indicate that TUBA4B can concurrently bind to and suppress miR-214 and miR-216a/b in GC.

**Fig. 4:** TUBA4B acts as a sponge for miR-214, miR-216a and miR-216b. **a** qRT-PCR analysis of the nuclear and cytoplasmic TUBA4B expression in MGC-803 and HGC-27 cells. **b** miRCode and miRWalk online database analysis for miRNAs that might bind to both TUBA4B and PTEN 3′-UTR. **c** RNA pull-down assay for measuring the interaction between TUBA4B and the indicated eight miRNAs in MGC-803 and HGC-27 cells. **d**–**f** Luciferase reporter assay in MGC-803 and HGC-27 cells co-transfected with wild-type or mutant TUBA4B reporter and control or miR-214/216a/b mimics. **g**, **h** qRT-PCR analysis of TUBA4B expression in GC cells and xenograft model after TUBA4B overexpression. **i** The Kaplan–Meier survival curve of GC patients with low and high miR-214, miR-216a and miR-216b expression in KM-plotter online database. *p < 0.05, **p < 0.01

### Identification of TUBA4B/miR-214/216a/b/PTEN/PI3K/AKT axis in GC

Subsequently, we tested whether miR-214 and miR-216a/b could target PTEN. As shown in Fig. 5a–c, overexpressed miR-214 or miR-216a/b significantly reduced the luciferase activity of PTEN 3′-UTR reporter vector containing wild-type miR-214 or miR-216a/b binding site, while had no effect on the mutated one. Further, exogenous expression of miR-214 or miR-216a/b dramatically decreased PTEN expression, whereas these reductions were completely blocked by overexpression of TUBA4B with wild-type miR-214 or miR-216a/b binding site, but not by overexpression of the mutant one (Fig. 5d–f). Functionally, about threefold increased proliferative capacities were observed in MGC-803 and HGC-27 cells overexpressing miR-214 or miR-216a/b compared with control cells (Fig. 5g–i), however, these enhanced proliferation effects were counteracted by TUBA4B overexpression or LY294002 treatment (a PI3K/AKT pathway inhibitor) (Fig. 5g–i). Altogether, the above results suggest that miR-214 and miR-216a/b mediate the regulation of TUBA4B on PTEN/PI3K/AKT signaling pathway.

**Fig. 5:** miR-214 and miR-216a/b mediate the regulation of TUBA4B on PTEN/PI3K/AKT signaling pathway. **a**–**c** Luciferase reporter assay in MGC-803 and HGC-27 cells co-transfected with wild-type or mutant PTEN 3′-UTR reporter and control or miR-214/216a/b mimics. **d**, **e** qRT-PCR analysis of PTEN expression in MGC-803 and HGC-27 cells co-transfected with control or miR-214/216a/b mimics and wild-type or mutant TUBA4B expression vector. **g**–**i** CCK-8 proliferative assay in MGC-803 and HGC-27 cells treated with control or miR-214/216a/b mimics and TUBA4B expression vector or LY294002. **j** The cartoon sketch showing the mechanism of the suppressive role of TUBA4B in GC, in which TUBA4B could abundantly sponge miR-214 and 216a/b to increase PTEN expression, leading to inactivation of oncogenic PI3K/AKT signaling, thus impeding GC aggressive progression. **p < 0.01

## Discussion

It has been well documented that lncRNA is linked to human diseases, including cancer [14]. Recently, a novel lncRNA, TUBA4B, was reported to be significantly decreased in breast cancer [15], non-small cell lung cancer [16] and ovarian cancer [17]. However, an in-depth study on its clinical significance and biological function in GC has never been undertaken. Here, we found that TUBA4B was also dramatically downregulated in GC tissues, cells and plasma, which was closely related to malignant clinicopathological features and adverse prognosis. Further studies revealed that TUBA4B was able to abundantly sponge miR-214 and miR-216a/b and upregulate PTEN expression, resulting in dampening oncogenic PI3K/AKT signaling, thereby retarding GC tumorigenesis and aggressiveness (Fig. 5j). Thus, our findings advance the understanding of TUBA4B in human cancers, and demonstrate that TUBA4B is also a anti-tumor factor in GC.

Up to now, numerous studies show that lncRNA is frequently dysregulated in human cancers and can be used as an effective biomarker [18]. For instance, high lncRNA SNHG1 expression was positively correlated with poor outcome in colorectal cancer patients [19]. LncRNA MALAT-1 expression in serum was identified as a good distinction between hepatocellular carcinoma patients and healthy controls [20]. LncRNA CASC11 was shown to be markedly increased in osteosarcoma and predicted dismal survival [21]. Likewise, some lncRNAs related to the diagnosis or prognosis of GC have been reported, such as FLJ22763 [22], GMAN [23], ZEB1-AS1 [24] and UCA1 [25]. Herein, we found that GC patients with low TUBA4B expression displayed shorter survival time than patients with high TUBA4B expression, and the AUC value based on plasma TUBA4B expression was 0.8075 (95% CI 0.7103 to 0.9047), implying that TUBA4B is an efficacious diagnostic and prognostic biomarker for GC patients. Further large sample studies are needed to confirm our findings, and it would be worthwhile to clarify the crosstalk between TUBA4B and the above reported GC-associated lncRNAs, and whether TUBA4B can be detected in urine and exosomes.

Accumulating evidence suggests that cytoplasmic lncRNA is capable of altering gene expression via directly interaction with miRNAs, a mechanism known as ceRNA [26]. Concordantly, by performing luciferase reporter and RNA pull-down assays, we identified that cytoplasmic TUBA4B could serve as an effective sponge for endogenous miR-214, miR-216a and miR-216b in GC cells. Several studies have reported that miR-214 was significantly upregulated in various cancers, including GC [27–29]. However, miR-216a and miR-216b were proposed to be the tumor suppressors in some solid tumors [30, 31], and the roles of these two miRNAs in GC remain unexplored. In this study, we found that TUBA4B overexpression dramatically reduced the expression of miR-216a and miR-216b, and GC patients with high miR-216a/b expression had worse prognosis than those with low miR-216a/b expression (survival data from Kaplan–Meier plotter database), hinting that miR-216a and miR-216b, like miR-214, are both oncogenes in GC. This notion was also confirmed by subsequent investigation that miR-214 and miR-216a/b could target the 3′-UTR of the well-known tumor suppressor PTEN and inhibit its expression, revealing that miR-214 and miR-216a/b are the mediators of TUBA4B and PTEN. It is widely accepted that PTEN is pervasively decreased in a various of human cancers and most oncogenic phenotypes caused by PTEN loss are attributed to the activation of PI3K/AKT signaling [32]. In our study, ectopic expression of TUBA4B remarkably increased PTEN expression and decreased p-PI3K and p-AKT expression, and the TUBA4B-induced attenuated aggressive phenotype was significantly rescued by PTEN silencing and AKT activator, suggesting PTEN/PI3K/AKT signaling is responsible for the function of TUBA4B. In all, these above findings indicate that TUBA4B functions as a pivotal negative regulator in GC progression mainly through dampening oncogenic PI3K/AKT pathway via alleviating the inhibitory effect of miR-214 and miR-216a/b on PTEN. Further study is warranted to explore the role of TUBA4B in other cancers. It is noteworthy that nearly 20% of TUBA4B were located in the nucleus. Emerging evidence demonstrates that nuclear lncRNA can modulate gene expression at the transcriptional level via recruiting some key proteins to the promoter regions [33, 34], it will be interesting to elucidate whether nuclear TUBA4B can also regulate PTEN expression through this mechanism.

## Conclusion

Our study for the first time suggests that TUBA4B is a tumor suppressor as well as a promising biomarker in GC. Restoration of TUBA4B may be a feasible therapeutic strategy against this thorny disease.

## Additional file

**Additional file 1: Figure S1.** FISH assay showing the cytoplasmic localization of TUBA4B. Nuclear was stained with DAPI.

## Data Availability

Please contact authors for data request.

## Abbreviations

lncRNA: long non-coding RNA
GC: gastric cancer
ceRNA: competitive endogenous RNA
TUBA4B: Tubulin Alpha 4B
CCK-8: Cell Counting Kit-8
